# Assessing forest fragmentation due to land use changes from 1992 to 2023: A spatio-temporal analysis using remote sensing data

**DOI:** 10.1016/j.heliyon.2024.e34710

**Published:** 2024-07-16

**Authors:** Khadim Hussain, Kaleem Mehmood, Shoaib Ahmad Anees, Zhidan Ding, Sultan Muhammad, Tariq Badshah, Fahad Shahzad, Ijlal Haidar, Abdul Wahab, Jamshid Ali, Mohammad Javed Ansari, Saleh H. Salmen, Sun Yujun, Waseem Razzaq Khan

**Affiliations:** a State Forestry and Grassland Administration Key Laboratory of Forest Resources and Environmental Management, Beijing Forestry University, Beijing, 100083, China; b Key Laboratory for Silviculture and Conservation of Ministry of Education, Beijing Forestry University, Beijing, 100083, China; c Institute of Forest Science, University of Swat, Main Campus Charbagh 19120, Swat, Pakistan; d Department of Forestry, The University of Agriculture, Dera Ismail Khan, 29050, Pakistan; e Key Laboratory of Environment Change and Resources Use in Beibu Gulf, Ministry of Education, Nanning Normal University, Nanning, 530001, China; f Department of Forestry and Wildlife, Faculty of Physical & Applied Sciences, University of Haripur, Pakistan; g Mapping and 3S Technology Center, Beijing Forestry University, Beijing, 100083, China; h Department of Forestry and Range Management, Arid Agriculture University Rawalpindi, Pakistan; i Department of Botany, Hindu College Moradabad (Mahatma Jyotiba Phule Rohilkhand University Bareilly), 244001, India; j Department of Botany and Microbiology, College of Science, King Saud University, PO Box -2455, Riyadh, 11451, Saudi Arabia; k Department of Forestry Science and Biodiversity, Faculty of Forestry and Environment, Universiti Putra Malaysia UPM, Serdang, 43400, Selangor, Malaysia; l Advanced Master in Sustainable Blue Economy, National Institute of Oceanography and Applied Geophysics - OGS, University of Trieste, Trieste, 34127, Italy; m Institut Ekosains Borneo (IEB), Universiti Putra Malaysia Bintulu Campus, Sarawak, 97008, Malaysia

**Keywords:** Remote sensing, Forest fragmentation, Spatial analysis, Land use change, Ecosystem services

## Abstract

The increasing pressures of urban development and agricultural expansion have significant implications for land use and land cover (LULC) dynamics, particularly in ecologically sensitive regions like the Murree and Kotli Sattian tehsils of the Rawalpindi district in Pakistan. This study's primary objective is to assess spatial variations within each LULC category over three decades (1992–2023) using cross-tabulation in ArcGIS to identify changes in LULC and investigates into forest fragmentation analysis using the Landscape Fragmentation Tool (LFTv2.0) to classify forest into several classes such as patch, edge, perforated, small core, medium core, and large core. Utilizing remote sensing data from Landsat 5 and Landsat 9 satellites, the research focuses on the temporal dynamics in various land classes including Coniferous Forest (CF), Evergreen Forest (EF), Arable Land (AR), Buildup Area (BU), Barren Land (BA), Water (WA), and Grassland (GL). The Support Vector Machine (SVM) classifier and ArcGIS software were employed for image processing and classification, ensuring accuracy in categorizing different land types. Our results indicate a notable reduction in forested areas, with Coniferous Forest (CF) decreasing from 363.9 km^2^, constituting 45.0 % of the area in 1992, to 291.5 km^2^ (36.0 %) in 2023, representing a total decrease of 72.4 km^2^. Similarly, Evergreen Forests have also seen a significant reduction, from 177.9 km^2^ (22.0 %) in 1992 to 99.8 km^2^ (12.3 %) in 2023, a decrease of 78.1 km^2^. The study investigates into forest fragmentation analysis using the Landscape Fragmentation Tool (LFTv2.0), revealing an increase in fragmentation and a decrease in large core forests from 20.3 % of the total area in 1992 to 7.2 % in 2023. Additionally, the patch forest area increased from 2.4 % in 1992 to 5.9 % in 2023, indicating significant fragmentation. Transition matrices and a Sankey diagram illustrate the transitions between different LULC classes, providing a comprehensive view of the dynamics of land-use changes and their implications for ecosystem services. These findings highlight the critical need for robust conservation strategies and effective land management practices. The study contributes to the understanding of LULC dynamics and forest fragmentation in the Himalayan region of Pakistan, offering insights essential for future land management and policymaking in the face of rapid environmental changes.

## 1 Introduction

Worldwide, forests and mountain ecosystems are undergoing substantial changes due to both natural processes [1] and human activities [[2], [3], [4], [5]]. There are many environmental consequences associated with changes in land cover, impacting biodiversity and global carbon and hydrologic cycles (K. [[6], [7], [8], [9]]). Over the past few decades, human activities and development have significantly driven Land Use and Land Cover Change (LULCC), interacting with natural environmental processes [[10], [11], [12], [13]]. This global transformation is closely linked to sustainable development [14]. Deforestation in Himalayan forests highlights significant environmental problems and has been the focus of intensive research [[15], [16], [17]]. The Himalayas of Pakistan, although acknowledged for their significant biodiversity, are experiencing increasing pressures on their forest cover due to human activities and natural factors, leading to rapid and extensive changes in land use cover (M. [[18], [19], [20]]). The region also faces risks such as landslides, heavy rainfall, floods, and forest fires, exacerbated by the fragile mountain terrain and ecosystems [[21], [22], [23], [24]]. If deforestation persists at the current rate, the world's total forest cover could be depleted within the next century, significantly contributing to climate change by reducing the capacity of forests to act as natural sinks for atmospheric carbon dioxide (CO_2_) [[25], [26], [27], [28], [29], [30]].

Forest fragmentation is another severe environmental issue with wide-ranging consequences for ecosystems and biodiversity globally ([]; T. U. [25,29]). This situation is particularly apparent in the Pakistan Himalayan Region, an area of rich biodiversity where the country faces critical vulnerabilities in conservation efforts ([31]; M. A. [32,33]). Forest fragmentation contributes to edge effects, resulting in changes in the physical structure and biological composition of ecosystems, affecting efficiency and species variety [[34], [35], [36], [37]]. Protected areas are crucial for the preservation of biodiversity. However, these areas face serious challenges such as forest fragmentation within their zones [[38], [39], [40]]. Enhancing habitat quality for species necessitates managing both protected areas and their buffer zones effectively to mitigate the negative effects of fragmentation [41,[42], [43], [44]]. Developing sustainable strategies requires a thorough understanding of the social, economic, cultural, and conservation aspects of forest fragmentation ([45]; K [6]).

The main goal of our research is to delve deeper into the complexities of forest fragmentation in the Indo-Himalaya region. Our objective is to thoroughly understand its underlying causes, impacts, and potential strategies for mitigation. The topography of Murree and Kotli Sattian Tehsils consists of rugged mountains, making direct ground monitoring challenging [46,47]. As a result, remote sensing and GIS tools are utilized to effectively analyze land use and forest fragmentation in these areas where direct observation is limited due to accessibility constraints. Analyzing changes in forested regions is critical for evaluating the effects of fragmented forests and shifts in LULC. This analysis holds significant importance for local planners, researchers, and the millions living within this region, including downstream communities [[46], [47], [48]]. Certain parts of our research area fall within the Margalla Hills Protected Area, introducing additional considerations for conservation purposes. Natural disturbances such as landslides, forest fires [24], and windthrows, alongside anthropogenic activities, have led to disruptions affecting forest cover and resulting in habitat fragmentation that supports diverse species [28,49]. Therefore, utilizing remote sensing (RS) and GIS methods for studying landscape changes and their environmental impacts is essential rather than optional.

## 2 Method

### 2.1 Study area context

Murree and Kotli Sattian, tehsils within the Rawalpindi district of Pakistan (33°47′15″ to 33°54′47″ N, 73°16′54″ to 73°29′18″ E), were selected for this study due to their unique ecological, hydrological, and topographical features. The region is predominantly covered by Chir Pine (Pinus roxburghii) forests, which are managed using the shelter-wood silviculture system. The Murree Forest Division (MFD) spans 47,285 acres, and Kotli Sattian covers 27,653 acres, both under the jurisdiction of the Punjab Forest Department. This extensive forested area is essential for studying silvicultural practices and biodiversity conservation. Kotli Sattian serves as a significant sub-watershed within the Indus and Jehlum River basins, highlighting its importance for watershed management research [49]. The study area's elevation ranges from 439 to 2274 m (Fig. 1), creating diverse altitudinal zones that support a variety of microclimates and rich biodiversity, which are crucial for ecological and climate impact studies. The region experiences temperatures ranging from −5 °C in winter to 40 °C in summer, with an annual precipitation of approximately 1140 mm, providing a unique setting to examine the effects of climate variability on forest ecosystems [50]. In addition to Chir Pine, the area is home to various species such as *Quercus incana* (rhin), *Pyrus pashia* (batangi), and *Pinus wallichiana* (kail), along with an understory consisting of *Dodonea viscosa* (sanatha), *Capparis decidua* (karir), *Adhatoda vasica (*Bahekar), *Cannabus sativa* (Bang), and *Berberis lycium* spp. (sumblu). This diverse vegetation composition facilitates studies on plant community dynamics and forest ecology [13].

**Fig. 1:** Map of the Study Area, Located in the Rawalpindi District of Pakistan. The Murree and Kotli Sattian Tehsils are the Study Area that Falls under Rawalpindi District.

The Murree and Kotli Sattian tehsils are representative of regions experiencing significant socio-economic and environmental pressures, including rapid urbanization, agricultural expansion, and infrastructure development. These pressures have led to prominent land use changes and forest fragmentation, similar to other ecologically sensitive regions worldwide. The study area's unique combination of ecological richness and socio-economic dynamics makes it an ideal case study for understanding the broader impacts of land use changes and forest fragmentation [5]. The findings from this study can be extrapolated to other mountainous and ecologically sensitive regions experiencing similar challenges. By providing valuable insights into the impacts of land use changes and forest fragmentation, this research offers a framework that can be applied to other regions with analogous socio-ecological contexts.

### 2.2 Data collection and pre-processing

This study predominantly utilizes remote sensing data derived from Landsat satellite imagery. The temporal scope of the analysis encompasses the years 1992, 2002, and 2012, utilizing Landsat 5 imagery sourced from the United States Geological Survey (USGS) https://earthexplorer.usgs.gov. For the year 2023, the investigation leveraged Landsat 9 imagery, also procured from the USGS. The geographical focus is defined by path 150 and row 36, ensuring a consistent study area across different periods. To maintain seasonal uniformity, data for all selected years were gathered during June. Shuttle Radar Topography Mission (SRTM) data was used in the derivation of the Digital Elevation Model (DEM). The DEM provides vital information about the vertical dimensions of the terrain. Also, the slope was calculated by using DEM data. Such categorization of the terrain into different height zones greatly enriches site analysis.

The utilization of these data sources significantly contributed to the visual interpretation of images, thereby ensuring accurate identification and categorization of land use. Both the Landsat TM and Landsat 8 OLI-TIRS sensors, as described in Table 1, provide a spatial resolution of 30 m, which is assumed sufficient for such analyses. Notably, Landsat imagery has demonstrated mapping accuracies exceeding 85 % across land use classes [51]. The integration of Landsat Operational Land Imager (OLI) with other data sources has further enhanced accuracy, achieving an impressive 98.62 % [52]. This underscores the pivotal role of Landsat imaging in land use classification. Prioritizing images without of clouds and shadows during selection was imperative to ensure the accuracy of land use categorization, as clouds significantly impact categorization precision [53]. Although imagery from different months was utilized throughout the investigation, our methodology was meticulously designed to uphold data quality and reliability.

**Table 1:** Description of landsat data acquired for the study.

Satellite	Sensor	Path/Row	Spatial Resolution (M)	Date of Acquisition	Sources
Landsat 5	TM	150/37,36	30	June 16, 1992	USGS
Landsat 5	TM	150/37,36	30	June 18, 2002	USGS
Landsat 5	TM	150/37,36	30	June 10, 2012	USGS
Landsat 9	OLI	150/37,36	30	June 10, 2023	USGS

In this study, we utilize ArcGIS Pro 3.1 and R programming for performing image processing tasks. ArcGIS is used for image processing and extracting vital information. The layer stacking method is employed to combine three particular bands into a single composite layer [54]. For Landsat 5 TM, bands 4, 3, and 2 are used, while bands 5, 4, and 3 are merged for Landsat 9 imagery [55]. Previous research has demonstrated that layer stacking is a powerful approach that can efficiently merge satellite imagery bands for tasks such as image enhancement and crop classification [56,57]. The study specifically investigates forest fragmentation, and a region of interest (ROI) is selected by overlaying the temporal images with the boundary and then extracting it. From the subset, fragmentation maps, as well as land use and land cover (LULC) maps, are generated. The study's region of Interest (ROI) was determined using the Universal Transverse Mercator (UTM) zone 42 N and resampled to achieve a 30-m spatial resolution. Accurate alignment of three different satellite images captured at different times was crucial to the study's success. To achieve this, 25 Ground Control Points (GCPs) were created throughout the study area. The Landsat-8 scene captured in 2023 was selected as the reference image for registration, with the study area situated at path 150 and rows 37 and 36. These images were then used to align the images acquired in 1992, 2002, and 2012 with the encouragement of a second-degree polynomial model for precise alignment (Afwani & Danoedoro, 2019; Eslami & Mohammadzadeh, 2015).

Atmospheric correction is a crucial step in the image processing pipeline for analyzing satellite data. The presence of gases, solid particles, and liquid particles in the atmosphere can distort satellite signals and affect the quality of data collected by the satellite. The radiance detected by the sensor called the Top of Atmosphere (TOA) radiance, can be significantly influenced by these atmospheric conditions. To rectify image distortions caused by atmospheric conditions, we used the technique proposed by Pahlevan et al. (2021) in combination with other studies (S. Kabir et al., 2020; Niraj et al., 2022). Atmospheric correction algorithms such as the 6 S model have been demonstrated to enhance the precision of satellite image analysis by considering factors like observational geometry, perspective angle, and weather conditions. (Martin et al., 2012). Studies have demonstrated that atmospheric correction reduces distorted signals and enhances the accuracy of data collected from satellite images (; H. Ma et al., 2015). Accurate determination of surface reflectance values requires corrections to eliminate atmospheric effects such as aerosol optical thickness. (AOT) (Hadjimitsis et al., 2010). The use of atmospheric correction and its integration into the overall image-processing workflow is illustrated in Fig. 2. It provides a full foundation of methodology.

**Fig. 2:** A comprehensive methodological procedure of the research.

### 2.3 Classification and analysis

Image analysis is crucial for identifying pixel groups with specific spectral characteristics and determining various land cover (LC) categories represented by these groups (Lambin and Geist, 2008). Image classification sorts pixels into distinct categories based on their spectral information, resulting in a thematic output. Landsat images were classified using support vector machine (SVM), known for its superior performance compared to traditional classifiers like Maximum Likelihood Estimation (Khatami et al., 2016).

SVM classifiers, based on statistical learning theory, minimize generalization error by finding a hyperplane that maximizes the margin between classes (Huang et al., 2002; Foody and Mathur, 2004; Pal and Mather, 2005). SVM aims to define a multidimensional space where class clusters are maximally separated, constructing a hyperplane using training data. Kernel methods transform non-linearly separable data into separable higher-dimensional space (Oommen et al., 2008; Candade and Dixon, 2004). Support vectors, crucial data points near the hyperplane, determine its position. The “C" parameter balances margin width and misclassification tolerance. SVRs offer versatility with regularization techniques and various kernel functions (Duda et al., 2016; Y. Li, Feng et al., 2020; Rodriguez-Galiano et al., 2015). SVM emerges as an efficient method, especially for non-linearly separable data.

For a two-class SVM, considering a training set *T* = {(x_1_, y_1_), ··· (x_1_, y_1_)} ∈ (*X* × Y)^*1*^, where ${\;x}_{i}\in$ X = $R^{n}$ and $y_{i}$ ∈ {1,−1} for (ⅈ = 1,2, …, l) representing the feature vector, the parameters C (consequence parameter) and the kernel function K ($x,x^{\prime }$) are predetermined (Eqs (1), (2))). The optimization problem is then formulated and resolved as follows [58].

(1) $$\begin{array}{c} \min_{\alpha }\frac{1}{2}\sum_{i=1}^{l}\sum_{j=1}^{l}y_{i\;}y_{j}\alpha_{i}\alpha_{j}\;K\left(x_{i}x_{j}\right)-\sum_{i=1}^{l}\alpha_{i}\; \end{array}$$

(2) $$\begin{array}{c} s.t.\;\sum_{i=1}^{l}y_{i}\alpha_{i}=0,0\leq \alpha_{i\;}\leq C,\dot{i}=1,\ldots ,l\; \end{array}$$

The optimal solution $\alpha^{*}={\left(\alpha^{*},\ldots ,\alpha^{*}\right)}^{T}$ is obtained. A positive component $\alpha^{*}:0\leq \alpha_{j}^{*}\leq C$ is then selected, and the threshold is computed as (Eq (3)) (Pang et al., 2022):

(3) $$\begin{array}{c} b^{*}=y_{j}-\sum_{i=1}^{1}y_{i\;}\alpha_{i}K\left(x_{i},x_{j}\right)\; \end{array}$$

Finally, the decision function is constructed in Eq (4):

(4) $$f\left(x\right)=sgn(\sum_{i=1}^{1}\;\alpha_{i}*y_{i\;}K\;\left(\;x,x_{i}\right)+b^{*}$$

### 2.4 Accuracy assessment and evaluation metrics

The model's performance for SVM was assessed using four key metrics: accuracy, precision, recall, and F1 score. These metrics provide a comprehensive evaluation of the model's ability to classify data accurately. Accuracy measures the ratio of correctly predicted instances to the total number of instances (including true positives and true negatives) [59]. It can be calculated using (Eq (5)).

(5) $$\text{Accuracy}=\frac{\text{TP}+\text{TN}}{\text{TP}+\text{TN}+\text{FP}+\text{FN}}$$

Where TP, TN, FP, and FN represent the number of true positives, the number of true negatives, false positives, and false negatives respectively.

Precision is the proportion of accurately predicted positive observations out of all predicted positive observations [[60], [61], [62]], as represented by (Eq (6)):

(6) $$\text{Precision}=\frac{\text{TP}+\text{FP}}{\text{TP}}$$

Recall (sensitivity) is determined by dividing properly predicted positive observations by the total actual class observations, as shown in (Eq (7)).

(7) $$\text{Recall}=\frac{\text{TP}+\text{FN}}{\text{TP}}$$

The F1 Score is computed as a balanced measure taking into account both precision and recall through their harmonic mean [63,64] in (Eq (8)).

(8) $$F1\;\text{Score}=2\times \frac{\text{Precision}\times \text{Recall}}{\text{Precision}+\text{Recall}}$$

To provide a more robust evaluation, we computed 95 % confidence intervals for the accuracy, precision, recall, and F1 score metrics. This was achieved using bootstrap resampling methods, which involved generating multiple bootstrap samples from the original data and calculating the performance metrics for each sample. The confidence intervals were then determined based on the distribution of these bootstrap results. Additionally, paired t-tests were conducted to evaluate the statistical significance of the differences in performance metrics between the years 1992, 2002, 2013, and 2023. This analysis helps to determine whether the observed improvements in the classification performance over the years are statistically significant. The paired t-tests compared the mean differences in accuracy, precision, recall, and F1 score between the different years, with a significance level set at p < 0.01. The results, including mean differences and p-values, are presented in the Results section. This enhanced methodology provides a more comprehensive understanding of the model's performance and the significance of improvements over time, ensuring the robustness and reliability of the classification results.

### 2.5 Forest fragmentation and change analysis

Satellite image categorization is a key process in change detection frameworks. These frameworks use time-based datasets to qualitatively evaluate the temporal evolution of different phenomena and measure the detected changes [65]. Change detection involves identifying differences in the state of an object or phenomenon by observing it at different points in time [66]. Our research entailed the examination of satellite information through a classification approach. This procedure categorized each image into seven classes. The classified classes are (i) Coniferous Forest, (ii) Evergreen Forest, (iii) Arable Land, (iv) Buildup Area, (v) Barren Land, (vi) Water, and (vii) Grassland. The categorization was performed using the Support Vector Machine model in R programming. This method has proven to be highly accurate and successful in numerous satellite image classification scenarios [67,68]. The criteria for classification are based on standard land use classification systems, similar to frameworks such as the Chinese Academy of Sciences land use classification. Table 2 of our study provides a comprehensive summary of the LULC categories identified during the classification process.

**Table 2:** Description of LULC classes.

LULC Classes	Description
**Coniferous Forest (CF)**	Land primarily covered with coniferous trees, characterized by a closed canopy.
**Evergreen Forest (EG)**	Areas with evergreen trees, including both scrub and open canopy forests.
**Arable Land (AR)**	Agricultural land used for crops, including cultivated fields and fallow land.
**Buildup Area (BU)**	Urbanized areas include residential, industrial, commercial zones, and transportation networks.
**Barren Land (BA)**	Landscapes with minimal vegetation, such as rocky areas and deserts.
**Water (WA)**	Bodies of water such as rivers, lakes, ponds, canals, and reservoirs.
**Grassland (GL)**	Areas dominated by grasses are not significantly disturbed by agricultural practices or urban development.

The research conducted an evaluation of spatial variations within each LULC classification over a span of thirty years. The analysis of LULC was facilitated through the utilization of a cross-tabulation module within the ArcGIS platform. The methodological approach employed is elucidated in Fig. 2, depicting a comprehensive matrix explaining changes in land use and land cover. This change matrix serves as a pivotal tool for acquiring detailed understandings into the characteristics and spatial distribution of alterations in land use [69]. As emphasized by Ma et al. [70], the significance of this approach lies in its ability to discern and quantify significant types or patterns of change within a designated research area. A detailed examination was undertaken to scrutinize variations in land use and land cover across specific time intervals: from 1992 to 2002, 2002 to 2013, and 2013 to 2023. During these periods, change matrices were employed to delineate alterations in land cover categories. Class gains were computed by subtracting the persistence value from the total row count, whereas losses were calculated by deducting the persistence value from the overall column total. The application of ArcGIS cross-tabulation for LULC change detection ensures a comprehensive understanding of the evolving patterns of land use and land cover [71,72].

The forest fragmentation assessment strategy employed the model developed by Vogt et al. [73], which characterized landscape fragmentation by analyzing image morphology. The analysis was facilitated through the Landscape Fragmentation Tool (LFTv2.0) provided by the University of Connecticut Centre for Land-use Education and Research. Operational within the ArcGIS environment, this tool required raster data, specifically land cover data categorized into non-forest and forest cover areas [74]. The LFT tool, an ArcGIS-based Toolbox, was readily deployable and facilitated the categorization of land cover maps into distinct classifications, including forest types such as Core, Edge, Patch, and Perforated. Within the core forest category, size-based distinctions were made, defining small core areas as those smaller than 1.00 km^2^, medium core areas as ranging between 1.00 and 2.00 km^2^, and large core areas as exceeding 2.00 km^2^ [75]. Evidence from studies by Forman & Deblinger [76] and Riitters et al. [77] underscored the presence and significance of the edge effect in influencing landscape fragmentation processes. In our study, an edge width of 100 m was incorporated, acknowledging potential variations based on the nature and extent of the study region. Previous research has demonstrated the efficacy of ArcGIS' LFT in evaluating forest fragmentation. For instance, in the north-western Himalaya, Sharma et al. (2017) observed that LFT accurately assessed forest fragmentation, revealing substantial landscape changes. Encisa-Garcia et al. [78] utilized LFT to examine forest fragmentation in the Baroro Waterway Watershed, revealing the decline of large forest regions and the expansion of smaller patches. These studies attest to the robustness and reliability of the tool's landscape fragmentation analysis, rendering it suitable for our investigation. These findings substantiate our methodology and offer a precise depiction of historical forest changes in the study area. The method proposed by Puyravaud [79] was employed in this study to calculate the annual rate of change for each LULC category, as well as the annual rate of pattern of forest fragments. Equation (9), widely recognized for its accuracy and simplicity, proved particularly valuable in assessing long-term changes in land cover studies.

(9) $$r=t_{2}-t_{1}\times \ln\left(A1A2\right)$$

Where *r* denotes the annual rate of change, *A*2 and *A*1 are the areas of the LULC class at the end and the beginning of the evaluated period, and *t* represents the number of years encompassing the period.

The approach has been used successfully in several studies to calculate yearly rates of change in land cover, including assessments of urban expansion, agricultural land alterations, and forest cover transition [[80], [81], [82]].The equation enabled our study to accurately quantify the elements of LULC changes and fragmentation in forestland, thereby offering vital information for natural resources management and the formulation of plans. This approach guarantees an in-depth understanding of the changing LULC patterns, as well as the allocation of forest fragmentation, throughout the selected periods.

## 3 Results

### 3.1 Temporal dynamics of Land Use and Land Cover Changes: a three-decade analysis (1992–2023)

The study explores the temporal analysis of anthropogenic and ecological changes in land use from 1992 to 2023, revealing a dynamic interplay throughout different classes. The land cover classes for 1992, 2002, 2013 and 2023 is shown in Fig. 3(A) and (B), 3(C), and 3(D) respectively. The Coniferous Forest (CF) was the dominant land classification in 1992, covering an area of 363.9 km^2^, which accounted for 45.0 % of the total land area. However, by 2023, its coverage had decreased to 291.5 km^2^, representing 36.0 % of the total land area. This trend is consistent with global urbanization diminishing forest cover [83]. The Evergreen Forest (EG) dropped from 177.9 km^2^ (22.0 %) in 1992 to 99.8 km^2^ (12.3 %) in 2023. The area of agricultural land (AL) expanded from 22.4 km^2^ (2.8 %) in 1992 to 82.9 km^2^ (10.2 %) in 2023, while the area of built-up land (BU) increased from 3.8 km^2^ (0.5 %) to 31.2 km^2^ (3.9 %). This indicates a worldwide pattern of urban and agricultural land trends, resulting in the expense of natural ecosystems [84]. Barren Land (BL) fluctuated from 27.2 km^2^ (3.4 %) to 20.2 km^2^ (2.5 %), then soared to 81.0 km^2^ (10.0 %) before another decrease to 21.0 km^2^ (2.6 %). Grass Land (GL) increased significantly from 209.5 km^2^ (25.9 %) to 279.5 km^2^ (34.5 %).

**Fig. 3:** LULC of 1992(A), 2002(B), 2013(C), and 2023(D).

Different land-use patterns are shown throughout each of the three time periods (1992–2002, 2002–2013, and 2013–2023). Between 1992 and 2002, there was a 21.6 km^2^ (2.7 % drop) in CF, an 8.6 km^2^ (1.1 %) increase in EG, and a 12.9 km^2^ (1.6 %) and 4.6 km^2^ (0.6 %) increase in AL and BU, respectively (Table 3). Between 2002 and 2013, there was an increase in AL and BU and a decrease in CF and EG. Forest areas continued to diminish from 2013 to 2023, whereas BU expanded while BL and GL fluctuated. These results demonstrate the complexity and dynamic character of land-use changes during the past 31 years (Fig. 3). Land-use class transitions, accompanied by quantitative area changes, indicate the intricate balance between natural biological processes and human-induced changes, guiding sustainable land management and policy development.

**Table 3:** Landcover area, percentage, change, and proportion of change in percentage.

Class Name	1992		2002		2013		2023		1992–2002		2002–2013		2013–2023	
	Area km^2^	%	Area km^2^	%	Area km^2^	%	Area km^2^	%	Km^2^	%	Km^2^	%	Km^2^	%
CF	363.9	45.0	342.3	42.3	305.0	37.7	291.5	36.0	−21.6	−2.7	−37.3	−4.6	−13.5	−1.6
EG	177.9	22.0	169.3	20.9	133.0	16.4	99.8	12.3	−8.6	−1.1	−36.3	−4.5	−33.2	−4.1
AL	22.4	2.8	35.3	4.4	80.0	9.9	82.9	10.2	12.9	1.6	44.7	5.5	2.9	0.4
BU	3.8	0.5	8.4	1.0	15.0	1.9	31.2	3.9	4.6	0.6	6.6	0.8	16.2	2.0
BL	27.2	3.4	20.2	2.5	81.0	10.0	21.0	2.6	−7.0	−0.9	60.8	7.5	−60.0	−7.4
WA	4.4	0.5	3.6	0.4	5.0	0.6	3.3	0.4	−0.8	−0.1	1.4	0.2	−1.7	−0.2
GL	209.5	25.9	230.1	28.4	191.0	23.6	279.5	34.5	20.6	2.6	−39.1	−4.9	88.5	11.0
**Total**	809.2	100.0	809.2	100.0	810.0	100.0	809.2	100.0						

### 3.2 Longitudinal performance analysis of SVM in supervised classification (1992–2023)

Support Vector Machines classifiers have been used for supervised classification over several years (1992, 2002, 2013, and 2023), providing valuable insights into the effectiveness of the model. By focusing on important metrics such as accuracy, precision, recall, and F1 score, a noticeable trend of ongoing improvement emerges.

In 2002, the model had an accuracy rate of 79.4 %, a precision rate of 87.07 %, a recall rate of 69.03 %, and an F1 score of 77.00 % as shown in Table 4. These statistics, especially the recall rate, indicated that there is potential for improvement in the model's capacity to reduce the number of false negatives. In 2013, ten years later, there was a significant enhancement in performance. The accuracy increased to 84.1 %, precision improved to 87.74 %, recall reached 79.26 %, and the F1 score was 83.28 %. This sequence demonstrates improvements in the model's ability to classify. In the studied period, the model reached its highest level of performance in 2023, with an accuracy of 87.0 %, a precision of 87.08 %, a recall of 87.28 %, and an F1 score of 87.18 %. The 2023 results demonstrate the model's robustness and reduced bias in classification, as evidenced by the balanced and high values in precision and recall. Interestingly, a retrospective study of the year 1992 shows the model with an accuracy of 81.7 %, a precision of 81.77 %, recall at 82.12 %, and an F1 score of 81.94 %, demonstrating that the model's earlier phases already had a relatively good basis in classification accuracy.

**Table 4:** Performance metrics of SVM-Based supervised classification model (1992–2023).

Year	Accuracy (%)	Precision (%)	Recall (%)	F1 Score (%)
1992	81.7	81.77	82.12	81.94
2002	79.4	87.07	69.03	77.00
2013	84.1	87.74	79.26	83.28
2023	87.0	87.08	87.28	87.18

The spatiotemporal study revealed an enhancement in the SVM-based model's capacity to accurately categorize data. The model's consistent high precision throughout the years demonstrates its reliability in accurately recognizing genuine positives. The upward trajectory of recall, particularly evident in the most recent data point from 2023, underscores the progressive improvement of the model in minimizing false negatives. Therefore, when the findings are merged with the independently generated Area Under the Curve (AUC) for each year shown in Fig. 4. They offer a complete insight of the model's overall performance and improvement in supervised classification tasks.

**Fig. 4:** Area under the curve (AUC) for each year.

### 3.3 Temporal analysis of SVM classification performance

The classification performance of the SVM model over the years 1992, 2002, 2013, and 2023 was assessed using Accuracy, Precision, Recall, and F1 Score metrics. The results, including 95 % confidence intervals, are presented in Fig. 5 (B). The accuracy of the SVM classification exhibited an overall increasing trend from 1992 to 2023. Initially, in 1992, the accuracy was approximately 81.7 % (CI: 80.1 %–83.3 %). However, there was a slight decrease in 2002 to approximately 79.4 % (CI: 77.8 %–81.0 %). From 2002 onwards, the accuracy showed a significant improvement, increasing to approximately 84.1 % in 2013 (CI: 82.6 %–85.6 %) and reaching 87.0 % in 2023 (CI: 85.6 %–88.4 %). Precision saw a notable improvement from 1992 to 2002, increasing from 81.77 % (CI: 80.3 %–83.2 %) to 87.07 % (CI: 85.6 %–88.5 %). It remained relatively stable with minor fluctuations, recording 87.74 % in 2013 (CI: 86.3 %–89.2 %) and 87.08 % in 2023 (CI: 85.3 %–89.7 %). Recall experienced a significant decrease from 82.12 % in 1992 (CI: 80.6 %–83.6 %) to 69.03 % in 2002 (CI: 67.1 %–71.0 %). However, it improved steadily in the subsequent years, increasing to 79.26 % in 2013 (CI: 77.5 %–81.0 %) and further to 87.28 % in 2023 (CI: 85.8 %–88.7 %). The F1 Score, which balances precision and recall, showed a decrease from 81.94 % in 1992 (CI: 80.5 %–83.4 %) to 77.00 % in 2002 (CI: 75.4 %–78.6 %). This was followed by an improvement to 83.28 % in 2013 (CI: 81.8 %–84.7 %) and further to 87.18 % in 2023 (CI: 85.7 %–88.6 %).

**Fig. 5:** (A) Trends of various metrics (Accuracy, Precision, Recall, and F1 Score) over the years 1992, 2002, 2013, and 2023. Each metric is represented with its mean value along with the corresponding confidence intervals. The metrics display variations and trends over time, highlighting the changes in performance. (B) Mean differences in metrics (Accuracy, Precision, Recall, and F1 Score) for paired comparisons between the years 1992, 2002, 2013, and 2023. The mean differences are shown with bars indicating significant differences (p < 0.01), providing insights into the statistical significance of changes in metrics over the specified time periods.

To evaluate the statistical significance of these changes, paired t-tests were conducted comparing the metrics between different years (1992 vs. 2002, 2002 vs. 2013, and 2013 vs. 2023), as shown in Fig. 5 (A). The results indicated a significant decrease in accuracy from 1992 to 2002, with a mean difference of 0.0234 (p < 0.01), followed by significant improvements from 2002 to 2023, with mean differences of −0.0473 (p < 0.01) from 2002 to 2013 and -0.0287 (p < 0.01) from 2013 to 2023. Precision improved significantly from 1992 to 2002, with a mean difference of −0.0530 (p < 0.01). It then showed a slight decrease from 2002 to 2013, with a mean difference of −0.0061 (p < 0.01), and a slight improvement from 2013 to 2023, with a mean difference of 0.0067 (p < 0.01). Recall showed a significant drop from 1992 to 2002, with a mean difference of 0.1302 (p < 0.01). This was followed by steady improvements, with mean differences of −0.1024 (p < 0.01) from 2002 to 2013 and -0.0803 (p < 0.01) from 2013 to 2023. The F1 Score decreased from 1992 to 2002, with a mean difference of 0.0493 (p < 0.01), but improved significantly from 2002 to 2023, with mean differences of −0.0629 (p < 0.01) from 2002 to 2013 and -0.0391 (p < 0.01) from 2013 to 2023. Overall, the statistical tests indicate significant improvements in the SVM classification performance over the years, particularly from 2002 onwards, with all p-values being less than 0.01 (Fig. 5 (B)). These visualizations and statistical analyses provide a comprehensive understanding of the changes in classification performance metrics over time, highlighting significant improvements and the robustness of the classification methods used.

### 3.4 Decadal land-use transitions and ecosystem dynamics (1992–2023)

The study's land-use transition matrices delineate the nuanced alterations within the landscape over four distinct periods labeled as ‘a,’ ‘b,’ ‘c,’ and ‘d,’ each symbolizing a different temporal scale of analysis, as evidenced by the accompanying Sankey diagram and tabular data (Table 5). During the initial phase ‘a,’ spanning from 1992 to 2002, the matrices reveal that Agricultural Land (AL) expanded into adjacent land classes, notably Barren Land (BL) and Grass Land (GL) by 9.0 km^2^ and 7.1 km^2^ respectively, indicating a trend towards agricultural proliferation. Coniferous Forest (CF) exhibited a notable internal transition of 216.3 km^2^, implying retention or regrowth within the same class, while simultaneously, 45.5 km^2^ transitioned to GL, potentially signifying land-use change towards non-forested landscapes, as given in S1. In phase ‘b,’ representing the interval from 2002 to 2013, the matrices suggest a continuation of these trends, with CF and Evergreen Forest (EGF) undergoing significant internal transitions, 229.1 km^2^, and 59.3 km^2^ respectively. This period also saw an increase in transitions from Barren Land (BL) to Coniferous Forest (CF) by 31.3 km^2^, possibly indicating a reversion to forested conditions or effective reforestation initiatives. The transitions from AL to GL remained substantial, at 14.3 km^2^, reflecting ongoing agricultural expansion. The ‘c' phase, encompassing 2013 to 2023, showed an intensification of transitions, with 201.5 km^2^ of CF transitioning within itself, and a further 66.9 km^2^ to GL. This implies a dramatic change in the way that forest land is managed or how ecological succession occurs. Additionally, the BL to GL transition increased to 29.4 km^2^, highlighting a potential shift in land-use policy or natural recovery of vegetation.

**Table 5:** Shows transition of area (km^2^) between classes in each period from 1992 to 2002, 2002–2013, 2013–2023.

		AL	BL	BU	CF	EGF	GL	WA
AL	a	**9.0**	1.8	1.1	0.3	1.0	7.1	0.0
	b	**12.7**	4.6	1.6	5.5	2.4	14.3	0.0
	c	**19.2**	4.0	6.0	12.4	1.1	48.5	0.0
	d	**7.3**	0.6	2.6	0.1	0.0	9.5	0.0
BL	a	0.7	**4.3**	0.8	6.3	2.1	10.5	0.1
	b	3.4	**8.0**	2.1	1.8	1.3	6.3	0.3
	c	9.6	**8.8**	9.9	30.5	1.9	29.4	0.0
	d	1.3	**3.0**	3.2	7.9	1.1	8.4	0.1
BU	a	0.2	0.4	**0.6**	0.6	0.5	1.4	0.0
	b	1.7	1.8	**1.9**	0.5	0.1	2.1	0.3
	c	3.3	1.6	**5.6**	0.5	0.3	6.5	0.2
	d	0.6	0.2	**1.1**	0.4	0.1	1.3	0.0
CF	a	5.3	4.3	0.9	**216.3**	46.2	45.5	0.1
	b	15.2	31.3	2.0	**229.1**	65.5	32.3	0.4
	c	10.3	1.6	2.5	**201.5**	50.1	66.9	0.0
	d	14.2	6.7	7.4	**188.3**	35.5	66.3	0.1
EGF	a	2.3	1.9	0.4	57.8	**68.6**	27.8	0.0
	b	14.7	12.2	2.9	57.7	**59.3**	46.1	0.2
	c	5.2	1.4	1.2	46.8	**52.5**	43.3	0.0
	d	12.2	4.0	4.8	43.1	**45.7**	49.0	0.0
GL	a	15.2	5.5	2.5	17.9	35.1	**107.5**	0.1
	b	43.4	32.1	7.3	38.4	21.8	**108.2**	0.4
	c	46.9	6.9	10.0	27.4	6.8	**111.3**	0.0
	d	39.7	4.8	8.9	14.4	7.4	**108.6**	0.1
WA	a	0.0	0.3	0.3	0.1	0.0	0.4	**2.8**
	b	0.0	0.1	0.2	0.0	0.0	0.0	**3.7**
	c	0.1	0.4	0.5	0.4	0.0	0.2	**3.5**
	d	0.0	0.4	0.4	0.1	0.0	0.3	**2.6**

“a” represents the transition area matrix from 1992 to 2002, “b” represents the transition area matrix from 2002 to 2013, “c” represents the transition area matrix from 2013 to 2023, “d” represents the transition area matrix from 1992 to 2023, row represent “from classes” and column represent “to classes”.

Over the full temporal scope from 1992 to 2023, labeled as ‘d,’ the data exhibits a broader perspective on land-use dynamics. CF showed a substantial retention of the area with 188.3 km^2^ transitioning within itself, indicating resilience or regrowth. However, transitions from CF to GL (66.3 km^2^) and EGF to CF (35.5 km^2^) were also significant, demonstrating the long-term shifts between forested and non-forested land classes. This pattern highlights effective landscape management practices that have likely contributed to the reduction of fragmented habitats and the augmentation of larger, more continuous ecological cores. Moreover, the Sankey diagram (Fig. 7) illustrates complex interactions involving non-Forest areas, with noticeable transitions to and from Core areas. These flows could represent reforestation efforts, changes due to natural regeneration, or shifts due to anthropogenic influences such as urban development or agricultural expansion. The two-way flows between Non-Forest and Core areas emphasize the ongoing dynamic nature of land-use changes and highlight the challenges in maintaining ecological stability amidst human activity.

### 3.5 Temporal analysis of forest fragmentation dynamics in murree: a comparative study from 1992 to 2023

The temporal dynamics of forest fragmentation in Murree were systematically analyzed utilizing ArcGIS Landscape Fragmentation Tool (LFT) version 2.0. This analysis provided critical insights into the spatial and temporal patterns of forest cover changes over the periods 1992, 2002, 2013, and 2023, as detailed in Table 6 and visually represented in Fig. 6(A) and (B), 6(C) and 6(D) respectively. A significant transformation in forest fragmentation patterns was observed across these intervals. In 1992, a predominant feature was the large core forest area (>202.343 ha), accounting for 20.3 % of the total study area. This was accompanied by 17.7 % edge forest, 20.2 % perforated forest, 2.4 % patch, and smaller percentages of small core (<101.17 ha) and medium core (101.17–202.34 ha) forests. By 2002, notable shifts were evident: the large core area experienced a 6.8 % decrease (from 164.3 to 109.5 km^2^), while the edge forest expanded by 2.2 % (from 143.5 to 161.3 ha). Concurrently, areas classified as patch, medium core, and small core underwent reductions of 3.3 % (from 19.2 to 45.7 km^2^), 1.5 % (from 15.2 to 27.4 km^2^), and 1.6 % (from 35.8 to 48.8 km^2^), respectively. The perforated area also increased by 1.6 % (from 162.5 to 176.1 km^2^). Notably, a 3.3 % overall decrease in non-forest areas from 1992 to 2002 suggested forest growth, yet the reduction in larger core areas indicated a degradation of protected forests in Murree.

**Table 6:** Forest fragmentation in area, percentage, and annual rate of change of each class.

	1992		2002		2013		2023		1992–2002		2002–2013		2013–2023	
Value	Area km2	%a	Area km2	%a	Area km2	%a	Area km2	%a	% Δ	%b	% Δ	%b	% Δ	%b
Non-Forest	267.6	33.1	240.5	29.7	326.7	40.3	377.1	46.6	−3.3	−1.0	10.6	3.6	6.3	1.5
Patch	19.3	2.4	45.7	5.6	67.8	8.4	48.1	5.9	3.3	13.6	2.7	4.9	−2.4	−2.9
Edge	143.5	17.7	161.3	19.9	176.8	21.8	158.3	19.6	2.2	1.2	1.9	1.0	−2.3	−1.0
Perforated	163.5	20.2	176.1	21.8	154.9	19.1	102.1	12.6	1.6	0.8	−2.6	−1.2	−6.5	−3.4
Core <250	35.8	4.4	48.8	6.0	51.8	6.4	48.2	6.0	1.6	3.6	0.4	0.6	−0.4	−0.7
Core 250–500	15.2	1.9	27.4	3.4	15.7	1.9	16.8	2.1	1.5	8.0	−1.5	−4.3	0.1	0.7
Core >500	164.3	20.3	109.5	13.5	16.3	2.0	58.6	7.2	−6.8	−3.3	−11.5	−8.5	5.2	25.9
Total	809.2	100.0	809.2	100.0	810.0	100	809.2	100						

a Percentage of each class out of the total area, % Δ = Percentage change in the component, %b Percentage of the annual rate of change in each class.

**Fig. 6:** Fragmentation classes for the years (a) 1992, (b) 2002, (c) 2013, and (d) 2023. The fragmentation classes include Patch, Edge, Perforated, Small Core, Medium Core, and Large Core. Part A (1992) shows the initial fragmentation patterns, Part B (2002) reflects changes due to land use dynamics over a decade, Part C (2013) highlights further fragmentation trends, and Part D (2023) illustrates the most recent fragmentation patterns, indicating significant increases in Patch and Edge areas and a notable decrease in Large Core areas.

**Fig. 7:** Sankey diagram represents flow of area between fragmentation classes in km^2^ from 1992 to 2023.

The subsequent interval from 2002 to 2013 revealed further changes: increases in patch, edge, and small core forest areas from 5.6 %, 19.9 %, and 6 % in 2002 to 8.4 %, 21.8 %, and 6.4 % in 2013, respectively. This period also saw a 2.7 %, 1.9 %, and 0.4 % component change, contrasted with 2.4 %, 2.3 %, and 0.40 % decreases in the following period. Drastic decreases of 11.5 % and 1.5 % in large and median core forests were recorded in 2013, followed by slight recoveries of 5.2 % and 0.1 % in 2023, respectively. The marked degradation of large core areas was attributed to forest fires. An increase in non-forest areas from 10.6 % in the second period to 6.3 % in the third period contrasted with a 3.3 % decrease in the first period. The annual rate of change for large core forests exhibited a declining trend of about 3.3 % and 11.5 % in the first (1992–2002) and second (2002–2013) periods, respectively, before rising to 25.9 % in the third period. This increase was partly attributed to initiatives like the BTTAP and other afforestation projects. Similarly, patch, edge, and small core forests displayed increasing annual rates of change in the first and second periods, whereas the medium core forest showed a decrease in the second period before increasing again in the first and third periods. The overall annual rate of change for total non-forest cover declined by 1.01 % in the first period and then increased from 3.58 % in the second period to 1.5 % in the third period.

### 3.6 Forest fragmentation and transitions from 1992 to 2023

The investigation carried out from 1992 to 2023 for landscape fragmentation provides a thorough comprehension of the development and alterations in forest cover. This study differentiates forest fragmentation into various categories such as Large Core, Medium Core, Small Core, Edge, and Perforated areas, and the area without forest is classified as non-forest class. The findings explore insights into significant trends and transitions to various classes as illustrated in tabular form (Table 7) and Fig. 7. It demonstrates the degree of forest degradation and the complex patterns of landscape transformation across time. There is a significant shift of 27.2 km^2^ from Large Core to Edge Forest. These major changes cause disturbances in fundamental habitats and the potential loss of biodiversity. Furthermore, the 35.9 km^2^ area of Large Core regions undergoes a shift into perforated landscapes, which stresses fragmentation vulnerability. This change is concerning because it may lead to a decline in habitat quality and an increase in edge effects. Furthermore, it would be detrimental to species that depend on the environmental circumstances found in the forest inland. Regardless of the Large Core Forest, the Medium Core is also undergoing significant shifts. More precisely, an area of 3.3 km^2^ transitions to Edge areas, and 2.4 km^2^ transforms into perforated landscapes highlighting the same pattern of fragmentation. Remarkably, areas surpassing 1.7 km^2^ transform into Large Core areas have positive potential for consolidation or expansion of habitats. These shifts illustrate the changing characteristics of forest landscapes and the adaptive boundaries that distinguish different forest classes. Although small core forest areas experience less change than larger core areas, they have significant effects on landscape dynamics. The key shift in transition highlights 6.2 km^2^ shifting to Perforated areas, 3.0 km^2^ converted to Patch areas, and 8.0 km^2^ persisting classified as Small Core. Forest fragmentation and landscape diversity are alternatively related to these changes in small cores in a broader context.

**Table 7:** Transition area matrix from 1992 (column) to 2023 (Row).

	Patch	Edge	Perforated	Small Core	Medium Core	Large Core	Non-forest	GT
Patch	3.7	1.4	0.2	0.0	0.0		14.0	19.3
Edge	15.2	45.3	6.3	2.8	0.5	0.8	72.6	143.4
Perforated	8.9	40.3	35.6	7.3	2.2	5.4	63.5	163.3
Small Core	3.0	8.3	6.2	8.0	0.6	0.5	9.0	35.7
Medium Core	0.5	3.3	2.4	3.0	1.7	0.7	3.7	15.2
Large Core	2.2	27.2	35.9	21.3	9.8	45.0	22.9	164.3
Non-forest	9.8	16.9	5.6	1.1	0.3	0.3	233.6	267.6
GT	43.2	142.7	92.2	43.5	15.1	52.8	419.4	808.9

This is critical to understand the pattern of the overall fragmentation process, it proposed careful investigation of the transition between classes like core forest to non-forest specifically from Large Core to Edge and Perforated classes. This trend highlights the need for immediate action to protect and restore forest ecosystems, as well as to implement effective land use planning strategies that prioritize conservation and sustainability. The alarming trend is evident in the significant rise of the non-forest category, which has increased from 267.6 km^2^ in 1992 to 419.4 km^2^ in 2023. This loss of forest cover has significant implications for ecosystem health and biodiversity conservation efforts. Furthermore, forest management practices need to prioritize the maintenance of ecological functions and biodiversity conservation to ensure the long-term sustainability of forest ecosystems. The study uncovers an elaborate and concerning pattern of transition in forest landscapes spanning three decades. By implementing effective conservation strategies, we can mitigate the negative impacts of agricultural expansion, urbanization, and climate change on biodiversity and natural ecosystems [85,86]. The alarming rate of deforestation and forest degradation necessitates urgent and comprehensive measures towards forest conservation and restoration.

### 3.7 Shifting landscape dynamics through tracking forest fragmentation

The fluctuations in the numbers of each land cover class over the past three decades indicate the dynamic nature of forest landscapes. In this case, the counts represent the number of counts in each class, the overall insight is given in Table 8. In 1992, the total count across all classes was 7,518, with the ‘Patch’ class having the highest count at 4034. This initial year shows a relatively balanced distribution among the classes, with ‘Small Core’ and ‘Perforated’ also having substantial counts. The overall number of counts in all categories in 1992 was 7,518, with the ‘Patch’ documenting the highest count at 4034. This initial year demonstrated an equal distribution across the different categories, as both ‘Small Core’ and ‘Perforated’ also had significant counts. By 2002, there was a significant rise in the overall count to 13,585, with the number of ‘Patch’ classes nearly doubling to 9873. This surge indicates a growth in smaller, fragmented forest regions. Other categories such as ‘Edge,’ ‘Perforated,’ and ‘Medium Core’ also showed growth, suggesting a shift towards increasingly fragmented environments. By 2013, the overall count had risen to 17,762, with ‘Patch’ remaining the most prevalent at 13,823. Nevertheless, there was a notable decline in the ‘Large Core’ category down to only 29, highlighting a concerned decrease in larger intact forest spaces. This year represents the highest in overall counts, indicating the intensified level of fragmentation compared to previous periods by 2023, the total count decreased to 11,107, with a reduction in the ‘Patch’ class to 8160. This decline across most categories may signify the consolidation of forest areas or changes in land use policies. However, the ‘Large Core’ category experienced a slight uptick to 71, potentially indicating some recovery or reclassification of forest areas. Table 7 depicts fluctuations in the quantities of different forest fragmentation categories from 1992 to 2023, totaling 49,972 counts over this period. The ‘Patch’ category shows the highest cumulative count 35,890. This notable rise over time within the ‘Patch’ class underscores the pattern towards increased forest fragmentation - an important concern for preserving biodiversity and managing ecosystems. The increase in counts within the ‘Patch’ category over time highlights a concerning tendency toward greater forest fragmentation that poses challenges for maintaining biodiversity and managing ecosystems. The variations in other categories, such as ‘Small Core,’ ‘Medium Core,’ and ‘Large Core,’ underscore the ever-changing characteristics of forest landscapes and the necessity for ongoing monitoring and flexible management approaches to mitigate the effects of fragmentation.

**Table 8:** Number of Counts in each class.

	Patch	Edge	Perforated	Small core	Medium Core	Large Core	Grand Total
1992	4034	160	1540	1548	24	212	7518
2002	9873	216	1753	1493	74	176	13,585
2013	13,823	280	1685	1901	44	29	17,762
2023	8160	203	1403	1215	55	71	11,107
Total	35,890	859	6381	6157	197	488	49,972

## 4 Discussion

The Temporal Changes in Land Use and Land Cover: An Analysis from 1992 to 2023″ highlights a significant shift in various land categories over three decades. The research illustrates the dynamic interaction between ecological changes and human influences. Coniferous Forest decreased from 363.9 km^2^ (45.0 %) in 1992 to 291.5 km^2^ (36.0 %) in 2023. Similarly, the Evergreen Forest experienced a decrease from its initial expanse of 177.9 km^2^ (22.0 %) in 1992 to just about half that size at 99.km^2^ (12.3 %), reflecting a pattern observed globally where urban development leads to the decline in forested regions. The study presents several innovative contributions to the field of remote sensing and land use analysis. Firstly, it offers a comprehensive longitudinal analysis over three decades (1992–2023), capturing long-term trends and patterns in land use and land cover (LULC) changes [87]. The integration of multiple remote sensing techniques, including data from Landsat 5 and Landsat 9, enhances the accuracy and detail of the assessment [88,89]. The use of the Support Vector Machine (SVM) classifier for image processing and classification demonstrates superior performance in handling complex and non-linear data relationships. Our classification results showed a high level of accuracy, with the overall accuracy improving from 79.4 % in 2002 to 87.0 % in 2023. The precision, recall, and F1 score metrics also demonstrated significant improvement over time, indicating the robustness and reliability of our classification approach [90]. Additionally, the application of the Landscape Fragmentation Tool (LFTv2.0) within ArcGIS for detailed forest fragmentation analysis provides nuanced insights into structural changes in forest landscapes. The integration of remote sensing data from multiple sources (Landsat 5 and Landsat 9) and advanced image processing techniques ensures a comprehensive and detailed analysis of land use and land cover (LULC) changes. Key steps such as atmospheric correction, layer stacking, and the use of the Landscape Fragmentation Tool (LFTv2.0) within ArcGIS contribute to the robustness of our methodology [91].

Our method is highly applicable to the study of forest fragmentation and land use changes in other ecologically sensitive regions. The approach can be effectively applied to analyze temporal and spatial patterns of land use changes in various landscapes, particularly those undergoing rapid urbanization and agricultural expansion. The detailed and accurate analysis provided by our methodology is crucial for informed decision-making and policy development. The study also incorporates comparative analyses with global studies, highlighting both common patterns and unique regional characteristics [92]. Finally, the research provides actionable insights for policymakers and conservationists, with recommendations for future land use management and conservation strategies, emphasizing the practical applications of the findings. By identifying specific areas of significant forest loss and fragmentation, our study provides actionable insights for developing targeted conservation strategies, reforestation projects, and sustainable land management practices. These efforts are essential for preserving biodiversity and maintaining ecosystem services [93]. The study has also highlighted considerable shifts in land use categories over three decades in Murree, with significant impacts on forest fragmentation and ecological balance. The decrease in Coniferous and Evergreen Forests is a global pattern exacerbated by urban development, like observations in Brazil and other global locations, which suggests a widespread environmental challenge of urban encroachment into forested areas [[94], [95], [96]]. Meanwhile, Agriculture Land (AL) expanded from 22.4 km^2^ (2.8 %) to 82.9 km^2^ (10.2 %), and Build-up Land (BU) increased from 3.8 km^2^ (0.5 %) to 31.2 km^2^ (3.9 %). The same result occurred in the study analyzed in Wenzhou City, China, where urbanization resulted in a reduction of forest areas and an expansion of urban environments [97]. In a parallel study from Jhelum District, Punjab, Pakistan, significant LULC were analyzed over a 30-year period, highlighting a considerable decrease in forest cover alongside increases in built-up areas due to urban expansion. The study also utilized NDVI and NDBI indices through remote sensing data to document these changes, providing a technical foundation that reinforces the findings from Murree (Majeed et al., 2021). Moreover, the changes in Barren Land and grassland correspond to alterations in other regions such as the San Juan Metropolitan Area, where the temperature response of vegetation is affected by urbanization [98]. The urban growth degrades the mangrove forest in Mumbai [95,99,100] representing the widespread occurrence of natural habitats being given up for urban expansion. This trend leads to an increase in the fragmentation of forests, resulting in biodiversity decline and degradation of ecosystems on a global scale [101,102]. The data indicates a corresponding increase in transition to counts within the ‘Patch’ and ‘Edge’ classes. This kind of fragmentation disturbs biological activities and contributes to the decline of ecosystem integrity, which has a negative effect on biodiversity and the health of forests [103,104]**.**

The process of forest fragmentation intensified as the substantial core forest experienced a notable reduction in size. An ongoing decline in the extensive primary forest and a rise in the fragmented forest signifies a rapid increase in forest fragmentation. The increase in the number of patches, small core, and medium core forests suggests that the forest is becoming increasingly disconnected from the major core forest area. The patch forest experienced a significant increase throughout the study period but was ultimately entirely degraded due to the edge effect [73]. The findings indicated a notable alteration in the large core forest because of the expansion of non-forest land. This leads to a loss of rare species that tolerate shade which is vital for maintaining ecological equilibrium [105]. The notable growth in the number of ‘Patch’ areas from 1992 to 2023, increasing from 4034 to 8,160, indicates an expansion of smaller and fragmented forest regions. This aligns with research suggesting that small forest fragments undergo significant structural changes, resulting in a decrease in biodiversity and degradation of ecosystems [106]. The overall increase in fragmentation, shown by the total count increasing from 7518 in 1992 to 11,107 in 2023, illustrates a worldwide trend where habitat fragmentation has significant effects on Earth's ecosystems. This decreases biodiversity and hinders crucial ecosystem functions [107]. The data indicates a changing landscape with important implications for conservation approaches and forest management aimed at lessening the impacts of fragmentation on biodiversity and ecosystem services.

While comparing our results with studies from the Himalayan region, similar trends were observed in forest fragmentation and deforestation. Mehmood et al. [75] assessed forest fragmentation in the Himalayan temperate region and reported a significant decrease in large forest cores alongside an increase in small core forests, reflecting our findings in Murree. Both studies employed the Landscape Fragmentation Tool (LFT v2.0) to demonstrate the substantial fragmentation driven by urbanization and anthropogenic activities. In the Garhwal Himalaya, Batar (2017) documented extensive deforestation and forest fragmentation over several decades, attributing these changes primarily to human activities. The patterns of deforestation and increased forest patches observed in the Garhwal Himalaya closely paralleled our results, highlighting the common impact of urbanization on forest ecosystems in both regions. Similarly, Qamer et al. [108] mapped deforestation in the Western Himalaya, revealing a loss of approximately 170,684 ha of forest over 20 years, equivalent to a 0.38 % annual deforestation rate. This aligned with the significant decline in forest cover identified in our study area, reflecting the persistent nature of deforestation in mountainous regions. Haq et al. [109] further supported our findings by highlighting the role of road networks and population growth in forest degradation within the Hindu Kush-Himalayan Mountains. Jamal [110] also studied deforestation rates in Murree using remote sensing, noting a 23 % decline in forest cover between 1999 and 2015, which reinforced the consistent trend of forest loss in the area. Ansari et al. [49] linked forest cover changes to climate variation in Murree, identifying a decrease in forest area by 8.26 % from 2001 to 2021 and correlating it with factors such as fuelwood collection, agriculture expansion, and urbanization. This integrated comparison emphasized the broader relevance of our findings, highlighting the similar socio-economic and environmental factors driving land use and forest cover changes across different mountainous regions, and underscored the need for region-specific conservation and land management strategies.

This study investigates the land-use and land-cover change patterns and their impacts on forest carbon dynamics around Islamabad and Rawalpindi using multispectral satellite images from 1990 to 2020. It provides valuable data on how urban expansion in these cities has influenced surrounding green areas, which could be comparable to the changes in Murree given the proximity and similar environmental pressures. Research shows that the unchecked urban expansion in Islamabad and Rawalpindi has led to significant decreases in forest areas and an increase in urban built-up areas, resulting in substantial changes in forest carbon storage [111]. The findings indicate a significant reduction in forest carbon stocks in Rawalpindi, while Islamabad showed some increase due to better forest management policies [112]. This suggests a broader regional environmental challenge related to urban encroachment into forested areas [113,114]. Human activity has led to the conversion of vegetation cover to non-forest areas, resulting in a rise in forest fragmentation. This poses a significant risk to biodiversity [4,12,115]. It is important to note that the growth in forest fragmentation is influenced by both natural and human factors (S. [4,5,116]). The findings of this study indicate that the primary factor contributing to forest fragmentation is the spread of agricultural and built-up areas. Additionally, the topography of the studied area has played a key influence in this process. Simultaneously, the research area exhibits a significant susceptibility to natural disasters, including major floods, landslides, and forest fires [24,117]. The forest is susceptible to alterations in its cover and an additional rise in fragmentation, which would further degrade the overall landscape of the forest. The reduction in forest area caused by the conversion to agriculture and other land uses, as well as the fragmentation of habitats, signifies a decline in available habitat [118]. Hence, overall alterations in forest fragmentation are expected to adversely affect the continuity and extent of forested land [119]. Forest fragmentation, along with changes in land cover, significantly affects biodiversity, resulting in habitat loss and a decline in ecosystem services within this region. The research on forest fragmentation in the Democratic Republic of Congo by Ref. [120] indicates an expansion in fragmentation over time, resulting in considerable biomass reduction [1], like the decline in large core forest regions noted in Murree. Furthermore, the arrangement of forest fragmentation can alter at various levels and is affected by the spatial scale or resolution of the landscape. Furthermore, the lower portion of the research area is designated as a protected area, affording it protected status. Nevertheless, the disturbance caused by ongoing human activities, such as road construction, migration of people to higher altitudes for farming, hydroelectric projects, and expansion of urban areas within the protected areas, poses a significant threat. These activities have the potential to disrupt the forest's continuity, diminish its magnitude, and impact connectivity, thereby reducing the overall forest land area.

## 5 Conclusions

The findings of this study underscore the complex dynamics of forest fragmentation and land use changes in the Murree and Kotli Sattian tehsils over the last three decades. The study reveals a marked decrease in core forest areas, with Coniferous Forests reducing from 363.9 km^2^ in 1992 to 291.5 km^2^ in 2023, and Evergreen Forests diminishing from 177.9 km^2^ to 99.8 km^2^ over the same period. These shifts indicate a substantial reduction of 19.9 % and 43.9 % in their respective areas, underlining the critical issue of forest degradation due to increasing urban and agricultural pressures. These trends show a significant decrease in core forest areas and increases in fragmented lands, highlighting the pressing need for targeted policy interventions and sustainable land management practices.

### 5.1 Policy implications

The study's results have important implications for land use policy and environmental management. The significant reduction in forest cover and increase in fragmentation call for immediate action to curb the encroachment of urban and agricultural development into forested lands. Effective policies are essential to protect remaining large core forests, promote reforestation, and mitigate further fragmentation.

### 5.2 Recommendations

Based on the findings of our study, we propose several practical recommendations for future land use management and conservation strategies to address the challenges identified. These recommendations are classified according to their relevancy and practicability.

• Implement zoning regulations that protect remaining large core forests and promote reforestation in highly fragmented regions.
• Develop and enforce stricter land use policies to prevent further deforestation and uncontrolled urban expansion.
• Promote agroforestry techniques and sustainable farming methods that minimize land degradation.
• Establish and expand protected areas to conserve critical habitats and biodiversity hotspots.
• Implement buffer zones around protected areas to mitigate the impact of human activities and promote ecological corridors.
• Engage local communities through education and awareness programs to highlight the importance of sustainable land use.
• Provide incentives for community-led forest conservation and sustainable agriculture initiatives.
• Develop capacity-building programs to train community members in sustainable land management practices.
• Establish long-term monitoring programs using remote sensing and GIS technologies to track changes in land use and forest fragmentation.
• Integrate policies aimed at reducing emissions from deforestation and forest degradation (REDD+) with local conservation strategies.

By implementing these recommendations, policymakers and land managers can develop effective strategies to mitigate the impacts of forest fragmentation, preserve biodiversity, and promote sustainable land use. The practical significance of our findings provides a valuable framework for guiding future land planning and conservation efforts in the Murree and Kotli Sattian tehsils and other regions facing similar socio-ecological challenges.

## Data and code availability

All references are mentioned in manuscript.

## Funding details

This research was funded by 10.13039/501100004530Universiti Putra Malaysia, Vote No. 9750500.

## CRediT authorship contribution statement

**Khadim Hussain:** Writing – review & editing, Writing – original draft, Visualization, Validation, Software, Methodology, Investigation, Formal analysis, Data curation, Conceptualization. **Kaleem Mehmood:** Writing – review & editing, Visualization, Software, Methodology, Investigation, Formal analysis. **Shoaib Ahmad Anees:** Writing – review & editing, Visualization, Software, Methodology, Investigation, Formal analysis. **Zhidan Ding:** Writing – review & editing. **Sultan Muhammad:** Writing – review & editing. **Tariq Badshah:** Writing – review & editing. **Fahad Shahzad:** Writing – review & editing. **Ijlal Haidar:** Writing – review & editing. **Abdul Wahab:** Writing – review & editing. **Jamshid Ali:** Writing – review & editing. **Mohammad Javed Ansari:** Writing – review & editing. **Saleh H. Salmen:** Writing – review & editing. **Sun Yujun:** Writing – review & editing, Supervision. **Waseem Razzaq Khan:** Writing – review & editing, Investigation, Formal analysis.

## Declaration of competing interest

The authors declare that they have no known competing financial interests or personal relationships that could have appeared to influence the work reported in this paper.

## References

[1] Luo M., Anees S.A., Huang Q., Qin X., Qin Z., Fan J., Han G., Zhang L., Shafri H.Z.M. (2024). Improving forest above-ground biomass estimation by integrating individual machine learning models. Forests.

[2] Foggin J.M. (2016).

[3] Prăvălie R. (2018). Major perturbations in the Earth's forest ecosystems. Possible implications for global warming. Earth Sci. Rev..

[4] Anees S.A., Zhang X., Khan K.A., Abbas M., Ghramh H.A., Ahmad Z. (2022). Estimation of fractional vegetation cover dynamics and its drivers based on multi-sensor data in Dera Ismail Khan, Pakistan. J. King Saud Univ. Sci..

[5] Anees S.A., Zhang X., Shakeel M., Al-Kahtani M.A., Khan K.A., Akram M., Ghramh H.A. (2022). Estimation of fractional vegetation cover dynamics based on satellite remote sensing in Pakistan: a comprehensive study on the FVC and its drivers. J. King Saud Univ. Sci..

[6] Sharma K., Robeson S.M., Thapa P., Saikia A. (2017). Land-use/land-cover change and forest fragmentation in the jigme dorji national park, Bhutan. Phys. Geogr..

[7] Singh A.K. (2021). Landscape fragmentation and land use and land cover analysis of the hinterland of ranchi: a case study of kanke block, 2001 and 2019. Urban India.

[8] Tuff K.T., Tuff T., Davies K.F. (2016). A framework for integrating thermal biology into fragmentation research. Ecol. Lett..

[9] Fopa V.K., Bayir N., Özdal D. (2023). Assessing the status and spatial-temporal dynamics of the bamenda mountains (BM), north west region of Cameroon. Environ. Monit. Assess..

[10] Regasa M.S., Nones M., Adeba D. (2021). A review on land use and land cover change in Ethiopian basins. Land.

[11] Aslam M.S., Huanxue P., Sohail S., Majeed M.T., Rahman S.U., Anees S.A. (2022). Assessment of major food crops production-based environmental efficiency in China, India, and Pakistan. Environ. Sci. Pollut. Control Ser..

[12] Mehmood K., Anees S.A., Luo M., Akram M., Zubair M., Khan K.A., Khan W.R. (2024). Assessing chilgoza pine (Pinus gerardiana) forest fire severity: remote sensing analysis, correlations, and predictive modeling for enhanced management strategies. Trees, Forests and People.

[13] Mehmood K., Anees S.A., Rehman A., Tariq A., Zubair M., Liu Q., Rabbi F., Khan K.A., Luo M. (2024). Exploring spatiotemporal dynamics of NDVI and climate-driven responses in ecosystems: insights for sustainable management and climate resilience. Ecol. Inf..

[14] Olorunfemi I.E., Fasinmirin J.T., Olufayo A.A., Komolafe A.A. (2020). GIS and remote sensing-based analysis of the impacts of land use/land cover change (LULCC) on the environmental sustainability of Ekiti State, southwestern Nigeria. Environ. Dev. Sustain..

[15] Dar A.A., Parthasarathy N. (2022). Patterns and drivers of tree carbon stocks in Kashmir Himalayan forests: implications for climate change mitigation. Ecological Processes.

[16] Ives J. (2004).

[17] Ullah S., Syed N.M., Gang T., Noor R.S., Ahmad S., Waqas M.M., Shah A.N., Ullah S. (2022). Recent global warming as a proximate cause of deforestation and forest degradation in northern Pakistan. PLoS One.

[18] Kabir M., Habiba U.E., Khan W., Shah A., Rahim S., Farooqi Z.U.R., Iqbal M.Z., Shafiq M. (2023).

[19] Muzaffarabad A.J. (2012). FISHERIES, ecology, wildlife, freshwater biology, marine biology. Zool. Soc. Pakistan Expresses Its Deep Gratitude to Vice Chancellor, Gov. Coll. Univ. Lahore, Pakistan Fac. Members Students Dep. Zool. Extending Warm Hosp.

[20] Nunes L.J.R., Meireles C.I.R., Pinto Gomes C.J., Almeida Ribeiro N.M.C. (2020). Forest contribution to climate change mitigation: management oriented to carbon capture and storage. Climate.

[21] Gordeeva E.M. (2021). Evolution of the international forest regulation. Kutafin Law Review.

[22] Miles Victoria, Esau Igor, Lasse Pettersson (2024). Using web GIS to promote stakeholder understanding of scientific results in sustainable urban development: A case study in Bergen, Norway. Sustain. Dev..

[23] Sohail M., Muhammad S., Mehmood K., Anees S.A., Rabbi F., Tayyab M., Hussain K., Hayat M., Khan U. (2023). Tourism, threat, and opportunities for the forest resources: a case study of gabin jabaa, district swat, khyber-pakhtunkhwa, Pakistan. Int. J. Forest Sci..

[24] Shahzad F., Mehmood K., Hussain K., Haidar I., Anees S.A., Muhammad S., Ali J., Adnan M., Wang Z., Feng Z. (2024). Comparing machine learning algorithms to predict vegetation fire detections in Pakistan. Fire Ecology.

[25] Nyaupane G.P., Chhetri N. (2009). Vulnerability to climate change of nature-based tourism in the Nepalese Himalayas. Tourism Geogr..

[26] Haider K., Khokhar M.F., Chishtie F., RazzaqKhan W., Hakeem K.R. (2017). Identification and future description of warming signatures over Pakistan with special emphasis on evolution of CO 2 levels and temperature during the first decade of the twenty-first century. Environ. Sci. Pollut. Control Ser..

[27] Jallat H., Khokhar M.F., Kudus K.A., Nazre M., Saqib N.U., Tahir U., Khan W.R. (2021). Monitoring carbon stock and land-use change in 5000-year-old juniper forest stand of Ziarat, Balochistan, through a synergistic approach. Forests.

[28] Khalid Noora (2019). A remotely sensed tracking of forest cover and associated temperature change in Margalla hills. Int. J. Digit. Earth.

[29] Khan T.U., Mannan A., Hacker C.E., Ahmad S., Amir Siddique M., Khan B.U., Din E.U., Chen M., Zhang C., Nizami M. (2021). Use of GIS and remote sensing data to understand the impacts of land use/land cover changes (LULCC) on snow leopard (Panthera uncia) habitat in Pakistan. Sustainability.

[30] Andreevich U.V., Reza S.S.O., Stepanovich T.I., Amirhossein A., Meng Z., Anees S.A., Petrovich C.V. (2020). Are there differences in the response of natural stand and plantation biomass to changes in temperature and precipitation? A case for two-needled pines in Eurasia. J. Resour. Ecol..

[31] Echeverría C., Coomes D., Salas J., Rey-Benayas J.M., Lara A., Newton A. (2006). Rapid deforestation and fragmentation of Chilean temperate forests. Biol. Conserv..

[32] Khan M.A., Khan M.A., Hussain M., Mujtaba G. (2014). Plant diversity and conservation status of himalayan region poonch valley azad kashmir (Pakistan). Pak. J. Pharm. Sci..

[33] Mehmood K., Anees S.A., Muhammad S., Hussain K., Shahzad F., Liu Q., Ansari M.J., Alharbi S.A., Khan W.R. (2024). Analyzing vegetation health dynamics across seasons and regions through NDVI and climatic variables. Sci. Rep..

[34] Carrara E., Arroyo-Rodríguez V., Vega-Rivera J.H., Schondube J.E., de Freitas S.M., Fahrig L. (2015). Impact of landscape composition and configuration on forest specialist and generalist bird species in the fragmented Lacandona rainforest, Mexico. Biol. Conserv..

[35] Joly C.A., Metzger J.P., Tabarelli M. (2014). Experiences from the B razilian A tlantic F orest: ecological findings and conservation initiatives. New Phytol..

[36] Rocha-Santos L., Pessoa M.S., Cassano C.R., Talora D.C., Orihuela R.L.L., Mariano-Neto E., Morante-Filho J.C., Faria D., Cazetta E. (2016). The shrinkage of a forest: landscape-scale deforestation leading to overall changes in local forest structure. Biol. Conserv..

[37] Taubert F., Fischer R., Groeneveld J., Lehmann S., Müller M.S., Rödig E., Wiegand T., Huth A. (2018). Global patterns of tropical forest fragmentation. Nature.

[38] Bingham H.C., Juffe Bignoli D., Lewis E., MacSharry B., Burgess N.D., Visconti P., Deguignet M., Misrachi M., Walpole M., Stewart J.L. (2019). Sixty years of tracking conservation progress using the World Database on Protected Areas. Nat. Ecol. & Evolution.

[39] Bingham H.C., Fitzsimons J.A., Mitchell B.A., Redford K.H., Stolton S. (2021). Privately protected areas: missing pieces of the global conservation puzzle. Front. Conserv. Sci..

[40] Pan S.A., Anees S.A., Li X., Yang X., Duan X., Li Z. (2023). Spatial and temporal patterns of non-structural carbohydrates in faxon fir (abies fargesii var. faxoniana), subalpine mountains of southwest China. Forests.

[41] de Moraes M.C.P., de Mello K., Toppa R.H. (2017). Protected areas and agricultural expansion: biodiversity conservation versus economic growth in the Southeast of Brazil. J. Environ. Manag..

[42] Nematollahi S., Fakheran S., Jafari A., Pourmanafi S., Kienast F. (2022). Applying a systematic conservation planning tool and ecological risk index for spatial prioritization and optimization of protected area networks in Iran. J. Nat. Conserv..

[43] Hussain K., Mehmood K., Yujun S., Badshah T., Anees S.A., Shahzad F., Nooruddin, Ali J., Bilal M. (2024). Analysing LULC transformations using remote sensing data: insights from a multilayer perceptron neural network approach. Spatial Sci..

[44] Li Y., Cai Y., Fu Q., Zhang X., Wan H., Yang Z. (2024). Dynamics of land use/land cover considering ecosystem services for a dense-population watershed based on a hybrid dual-subject agent and cellular automaton modeling approach. Engineering.

[45] Nagendra H., Pareeth S., Sharma B., Schweik C.M., Adhikari K.R. (2008). Forest fragmentation and regrowth in an institutional mosaic of community, government and private ownership in Nepal. Landsc. Ecol..

[46] Kausar R., Baig S., Riaz I. (2016). Spatio-temporal land use/land cover analysis of Murree using remote sensing and GIS. Asian J. Agric. Rural Dev. [En Línea].

[47] Tariq A., Shu H., Siddiqui S., Mousa B.G., Munir I., Nasri A., Waqas H., Lu L., Baqa M.F. (2021). Forest fire monitoring using spatial-statistical and Geo-spatial analysis of factors determining forest fire in Margalla Hills, Islamabad, Pakistan. Geomatics, Nat. Hazards Risk.

[48] Iqbal M.F., Khan I.A. (2014). Spatiotemporal land use land cover change analysis and erosion risk mapping of Azad Jammu and Kashmir, Pakistan. The Egyptian J. Rem. Sens. Space Sci..

[49] Ansari L., Ahmad W., Saleem A., Imran M., Malik K., Hussain I., Tariq H., Munir M. (2022). Forest cover change and climate variation in subtropical Chir pine forests of murree through GIS. Forests.

[50] Nizami S.M. (2012). The inventory of the carbon stocks in sub tropical forests of Pakistan for reporting under Kyoto Protocol. J. For. Res..

[51] Aitkenhead M.J., Aalders I.H. (2009). Predicting land cover using GIS, Bayesian and evolutionary algorithm methods. J. Environ. Manag..

[52] Sameen M.I., Nahhas F.H., Buraihi F.H., Pradhan B., Shariff A.R.B.M. (2016). A refined classification approach by integrating Landsat Operational Land Imager (OLI) and RADARSAT-2 imagery for land-use and land-cover mapping in a tropical area. Int. J. Rem. Sens..

[53] Cerbelaud A., Roupioz L., Blanchet G., Breil P., Briottet X. (2021). A repeatable change detection approach to map extreme storm-related damages caused by intense surface runoff based on optical and SAR remote sensing: evidence from three case studies in the South of France. ISPRS J. Photogrammetry Remote Sens..

[54] Pan X., Wang Z., Gao Y., Dang X., Han Y. (2022). Detailed and automated classification of land use/land cover using machine learning algorithms in Google Earth Engine. Geocarto Int..

[55] Al-Doski J., Mansor S.B., Ng H., San P., Khuzaimah Z. (2020). Land cover mapping using remote sensing data. Am. J. Geogr. Inf. Syst..

[56] Rivera A.J., Perez-Godoy M.D., Elizondo D., Deka L., del Jesus M.J. (2022). Analysis of clustering methods for crop type mapping using satellite imagery. Neurocomputing.

[57] Syrris V., Ferri S., Ehrlich D., Pesaresi M. (2015). Image enhancement and feature extraction based on low-resolution satellite data. IEEE J. Sel. Top. Appl. Earth Obs. Rem. Sens..

[58] Zhou T., Lu H., Wenwen W., Xia Y. (2019). GA-SVM based feature selection and parameter optimization in hospitalization expense modeling. Appl. Soft Comput..

[59] Tangirala S. (2020). Evaluating the impact of GINI index and information gain on classification using decision tree classifier algorithm. Int. J. Adv. Comput. Sci. Appl..

[60] Gnanvi J.E., Salako K.V., Kotanmi G.B., Kakaï R.G. (2021). On the reliability of predictions on Covid-19 dynamics: a systematic and critical review of modelling techniques. Infectious Disease Modell..

[61] Poldrack R.A., Huckins G., Varoquaux G. (2020). Establishment of best practices for evidence for prediction: a review. JAMA Psychiatr..

[62] Talukdar S., Singha P., Mahato S., Pal S., Liou Y.-A., Rahman A. (2020). Land-use land-cover classification by machine learning classifiers for satellite observations—a review. Rem. Sens..

[63] Chowdhury S., Schoen M.P. (2020). 2020 Intermountain Engineering, Technology and Computing (IETC).

[64] Yacouby R., Axman D. (2020). Proceedings of the First Workshop on Evaluation and Comparison of NLP Systems.

[65] Yu C., Liu B., Deng S., Li Z., Liu W., Ye D., Hu J., Peng X. (2023). Using medium-resolution remote sensing satellite images to evaluate recent changes and future development trends of mangrove forests on hainan island, China. Forests.

[66] Alawamy J.S., Balasundram S.K., Mohd Hanif A.H., Boon Sung C.T. (2020). Detecting and analyzing land use and land cover changes in the region of Al-Jabal Al-Akhdar, Libya using time-series landsat data from 1985 to 2017. Sustainability.

[67] Basheer S., Wang X., Farooque A.A., Nawaz R.A., Liu K., Adekanmbi T., Liu S. (2022). Comparison of land use land cover classifiers using different satellite imagery and machine learning techniques. Rem. Sens..

[68] Furuya M.T.G., Furuya D.E.G., Osco L.P., Ramos A.P.M. (2021). Classificação de superfícies impermeáveis em imagem multiespectral com algoritmo de machine learning. Colloquium Exactarum.

[69] Christensen M., Jokar Arsanjani J. (2020). Stimulating implementation of sustainable development goals and conservation action: predicting future land use/cover change in Virunga National Park, Congo. Sustainability.

[70] Ma S., Wang L.-J., Wang H.-Y., Zhao Y.-G., Jiang J. (2023). Impacts of land use/land cover and soil property changes on soil erosion in the black soil region, China. J. Environ. Manag..

[71] Mebrie D.W., Assefa T.T., Yimam A.Y., Belay S.A. (2023). A remote sensing approach to estimate variable crop coefficient and evapotranspiration for improved water productivity in the Ethiopian highlands. Appl. Water Sci..

[72] Ramanamurthy B.V., Vijayasaradhi B. (2021). Change detection analysis in LULC of the upstream Thandava reservoir using RS and GIS applications. IOP Conf. Ser. Mater. Sci. Eng..

[73] Vogt P., Riitters K.H., Estreguil C., Kozak J., Wade T.G., Wickham J.D. (2007). Mapping spatial patterns with morphological image processing. Landsc. Ecol..

[74] Parent J.R., Volin J.C. (2016). Validating Landsat-based landscape metrics with fine-grained land cover data. Ecol. Indicat..

[75] Mehmood K., Anees S.A., Rehman A., Tariq A., Liu Q., Muhammad S., Hatamleh W.A. (2024). Assessing forest cover changes and fragmentation in the Himalayan Temperate Region: implications for forest conservation and management. J. For. Res..

[76] Forman R.T.T., Deblinger R.D. (2000). The ecological road‐effect zone of a Massachusetts (USA) suburban highway. Conserv. Biol..

[77] Riitters K.H., Wickham J.D., Coulston J.W. (2004). A preliminary assessment of Montreal process indicators of forest fragmentation for the United States. Environ. Monit. Assess..

[78] Encisa-Garcia J., Pulhin J., Cruz R.V., Simondac-Peria A., Ramirez M.A., De Luna C. (2020). Land use/land cover changes assessment and forest fragmentation analysis in the Baroro river watershed, La union, Philippines. J. Environ. Sci. Manag..

[79] Puyravaud J.-P. (2003). Standardizing the calculation of the annual rate of deforestation. For. Ecol. Manag..

[80] Buraka T., Elias E., Lelago A. (2021). Southern Ethiopia.

[81] Hou A., Samuel A.B., Li M., Zheng Z., Xia J., Zhang X., Zhou G. (2020). Land use and land cover change of Ghana. IGARSS 2020-2020 IEEE Int. Geosci. Remote Sens. Symp..

[82] Melody S.M., Bennett E., Clifford H.D., Johnston F.H., Shepherd C.C.J., Alach Z., Lester M., Wood L.J., Franklin P., Zosky G.R. (2016). A cross-sectional survey of environmental health in remote Aboriginal communities in Western Australia. Int. J. Environ. Health Res..

[83] Lee C.M., Park J.W., Kwon T.-S., Kim S.-S., Ryu J.W., Jung S.J., Lee S.K. (2015). Diversity and density of butterfly communities in urban green areas: an analytical approach using GIS. Zool. Stud..

[84] Qi Z.-F., Ye X.-Y., Zhang H., Yu Z.-L. (2014). Land fragmentation and variation of ecosystem services in the context of rapid urbanization: the case of Taizhou city, China. Stoch. Environ. Res. Risk Assess..

[85] Shobairi S.O.R., Lin H., Usoltsev V.A., Osmirko A.A., Tsepordey I.S., Ye Z., Anees S.A. (2022). A comparative pattern for populus spp. and betula spp. stand biomass in eurasian climate gradients. Croat. J. For. Eng.: J. Theory and Appl. Forestry Eng..

[86] Anees S.A., Yang X., Mehmood K. (2024). The stoichiometric characteristics and the relationship with hydraulic and morphological traits of the Faxon fir in the subalpine coniferous forest of Southwest China. Ecol. Indicat..

[87] Santos M.J., Smith A.B., Dekker S.C., Eppinga M.B., Leitão P.J., Moreno-Mateos D., Morueta-Holme N., Ruggeri M. (2021). The role of land use and land cover change in climate change vulnerability assessments of biodiversity: a systematic review. Landsc. Ecol..

[88] Adepoju K.A., Adelabu S.A. (2020). Improving accuracy evaluation of Landsat-8 OLI using image composite and multisource data with Google Earth Engine. Remote Sens. Lett..

[89] Badshah M.T., Hussain K., Rehman A.U.R., Mehmood K., Muhammad B., Wiarta R., Silamon R.F., Khan M.A., Meng J. (2024). The role of random forest and Markov chain models in understanding metropolitan urban growth trajectory. Front. Forests and Glob. Change.

[90] Sheykhmousa M., Mahdianpari M., Ghanbari H., Mohammadimanesh F., Ghamisi P., Homayouni S. (2020). Support vector machine versus random forest for remote sensing image classification: a meta-analysis and systematic review. IEEE J. Sel. Top. Appl. Earth Obs. Rem. Sens..

[91] Fynn I.E.M., Campbell J. (2019). Forest fragmentation analysis from multiple imaging formats. J. Landscape Ecol.(Czech Republic).

[92] Winkler K., Fuchs R., Rounsevell M., Herold M. (2021). Global land use changes are four times greater than previously estimated. Nat. Commun..

[93] Kato S., Huang W. (2021). Land use management recommendations for reducing the risk of downstream flooding based on a land use change analysis and the concept of ecosystem-based disaster risk reduction. J. Environ. Manag..

[94] Sloan S., Sayer J.A. (2015). Forest Resources Assessment of 2015 shows positive global trends but forest loss and degradation persist in poor tropical countries. For. Ecol. Manag..

[95] Chouhan H.A., Parthasarathy D., Pattanaik S. (2018). 18 Coastal environmental vulnerability. Towards Coastal Resilience and Sustain..

[96] Baptista S.R., Rudel T.K. (2006). A re-emerging Atlantic forest? Urbanization, industrialization and the forest transition in Santa Catarina, southern Brazil. Environ. Conserv..

[97] Zhang X., Liao L., Xu Z., Zhang J., Chi M., Lan S., Gan Q. (2022). Interactive effects on habitat quality using InVEST and GeoDetector models in Wenzhou, China. Land.

[98] Comarazamy D.E., González J.E., Moshary F., Piasecki M. (2015). On the hydrometeorological changes of a tropical water basin in the Caribbean and its sensitivity to midterm changes in regional climate. J. Hydrometeorol..

[99] Khan W.R., Rasheed F., Zulkifli S.Z., Kasim M.R.B.M., Zimmer M., Pazi A.M., Kamrudin N.A., Zafar Z., Faridah-Hanum I., Nazre M. (2020). Phytoextraction potential of Rhizophora apiculata: a case study in Matang mangrove forest reserve, Malaysia. Trop. Conserv. Sci..

[100] Khan W.R., Nazre M., Akram S., Anees S.A., Mehmood K., Ibrahim F.H., Zhu X. (2024). Assessing the productivity of the matang mangrove forest reserve: review of one of the best-managed mangrove forests. Forests.

[101] Hanski I. (2011). Habitat loss, the dynamics of biodiversity, and a perspective on conservation. Ambio.

[102] Akram M., Hayat U., Shi J., Anees S.A. (2022). Association of the female flight ability of asian spongy moths (Lymantria dispar asiatica) with locality, age and mating: a case study from China. Forests.

[103] Devi A.R., Sudhakar Reddy C., Shimrah T. (2021). Assessment of forest fragmentation in a traditional shifting agricultural landscape in Senapati District of Manipur, Northeast India. Environ. Dev. Sustain..

[104] Muhammad S., Mehmood K., Anees S.A., Tayyab M., Rabbi F., Hussain K., Rahman H.U., Hayat M., Khan U. (2023). Assessment of regeneration response of silver fir (abies pindrow) to slope, aspect, and altitude in miandam area in district swat, khyber-pakhtunkhwa, Pakistan. Int. J. Forest Sci..

[105] Hill J.L., Curran P.J. (2001). Species composition in fragmented forests: conservation implications of changing forest area. Appl. Geogr..

[106] Pütz S., Groeneveld J., Alves L.F., Metzger J.P., Huth A. (2011). Fragmentation drives tropical forest fragments to early successional states: a modelling study for Brazilian Atlantic forests. Ecol. Model..

[107] Haddad N.M., Brudvig L.A., Clobert J., Davies K.F., Gonzalez A., Holt R.D., Lovejoy T.E., Sexton J.O., Austin M.P., Collins C.D. (2015). Habitat fragmentation and its lasting impact on Earth's ecosystems. Sci. Adv..

[108] Qamer F.M., Shehzad K., Abbas S., Murthy M.S.R., Xi C., Gilani H., Bajracharya B. (2016). Mapping deforestation and forest degradation patterns in western Himalaya, Pakistan. Rem. Sens..

[109] Haq N.u., Haq F., Rahman F. (2022). Extension of roads towards forest in palas valley Indus kohistan, Hindu kush-himalayan mountains, Pakistan. Geojournal.

[110] Jamal T., Naseer S., Hassan S.S., Batool H., Mahmood R., Naz A., Ali A. (2018). Appraisal of deforestation in Murree through open source satellite imagery. Adv. Rem. Sens..

[111] Hassan Z., Shabbir R., Ahmad S.S., Malik A.H., Aziz N., Butt A., Erum S. (2016). Dynamics of land use and land cover change (LULCC) using geospatial techniques: a case study of Islamabad Pakistan. SpringerPlus.

[112] Mannan A., Yongxiang F., Khan T.U., Nizami S.M., Mukete B., Ahmad A., Amara U., Liu J., Wali Muhammad M. (2021). Urban growth patterns and forest carbon dynamics in the metropolitan twin cities of Islamabad and Rawalpindi, Pakistan. Sustainability.

[113] Usoltsev V.A., Chen B., Shobairi S.O.R., Tsepordey I.S., Chasovskikh V.P., Anees S.A. (2020). Patterns for Populus spp. stand biomass in gradients of winter temperature and precipitation of Eurasia. Forests.

[114] Usoltsev V.A., Lin H., Shobairi S.O.R., Tsepordey I.S., Ye Z., Anees S.A. (2022). The principle of space-for-time substitution in predicting Betula spp. Biomass change related to climate shifts. Appl. Ecol. Environ. Res..

[115] Batar A.K., Watanabe T., Kumar A. (2017). Assessment of land-use/land-cover change and forest fragmentation in the Garhwal Himalayan Region of India. Environments.

[116] Sharma S., Roy P.S. (2007). Forest fragmentation in the Himalaya: a central himalayan case study. Int. J. Sustain. Dev. World Ecol..

[117] Tariq A., Shu H. (2020). CA-Markov chain analysis of seasonal land surface temperature and land use landcover change using optical multi-temporal satellite data of Faisalabad, Pakistan. Rem. Sens..

[118] Munsi M., Malaviya S., Oinam G., Joshi P.K. (2010). A landscape approach for quantifying land-use and land-cover change (1976–2006) in middle Himalaya. Reg. Environ. Change.

[119] Zomer R.J., Ustin S.L., Carpenter C.C. (2001). Land cover change along tropical and subtropical riparian corridors within the makalu barun national park and conservation area, Nepal. Mt. Res. Dev..

[120] Shapiro A.C., Aguilar-Amuchastegui N., Hostert P., Bastin J.-F. (2016). Using fragmentation to assess degradation of forest edges in Democratic Republic of Congo. Carbon Bal. Manag..

